RETRACTED

# Decreased miR-204 in H. pylori-Associated Gastric Cancer Promotes Cancer Cell Proliferation and Invasion by Targeting SOX4

**DOI:** 10.1371/journal.pone.0101457

**Published:** 2014-07-01

**Authors:** Xiaoying Zhou, Lin Li, Jing Su, Guoxin Zhang

**Affiliations:** 1 Department of Gastroenterology, First Affiliated Hospital of Nanjing Medical University, Nanjing, China; 2 First Clinical Medical College of Nanjing Medical University, Nanjing, China; H.Lee Moffitt Cancer Center & Research Institute, United States of America

## Abstract

**Background:**

The molecular mechanism between Helicobacter pylori (H. pylori) infection and gastric cancer remained largely unknown. In this study, we determined the role of miRNA in H. pylori induced gastric cancer.

**Methods and Results:**

We found that miR-204 was decreased in H. pylori positive tissues by qRT-PCR. Knockdown of miR-204 enhanced the invasion and proliferation ability of gastric cancer cells in vitro. Luciferase assay revealed that SOX4 was target gene of miR-204, which was found up-regulated in H. pylori positive tissues. Down-regulation of miR-204 and over-expression of SOX4 promoted epithelial-mesenchymal transition process.

**Conclusion:**

Taken together, our findings demonstrated that miR-204 may act as a tumor suppressor in H. pylori induced gastric cancer by targeting SOX4.

## Introduction

Gastric cancer is the fourth most common cancer and second leading cause of cancer-related death worldwide [1]. To date, molecular mechanisms on gastric cancer have been investigated, however, they have not fully understood [2]. Gastric carcinomas are supposed to develop according to a multistep process of carcinogenesis, which is strongly associated with the infection by the bacterial pathogen, *Helicobacter pylori*(*H. pylori*) [3]. *H. pylori*, which colonizes the stomach of 50% of the world population, has been classified as a class I carcinogen because of its causative role in the development of gastric cancer [4].

It has been reported that the development and progression of gastric cancer may be attributed to microRNAs (miRNAs) [5]–[8]. MiRNAs are small, non-coding RNAs that regulate the expression of target genes through translational repression or messenger RNA (mRNA) degradation [9]. MiR-204 aberrant expression was reported to associate with various cancers [10], [11]. However, little is known about miRNA-204 function in gastric cancer. Matsushima performed miRNA array study in H. pylori positive tissues and contols and found that miR-204 expression was significantly lower in H. pylori positive tissues [12].

In humans, the sex-determining region Y (SRY) box family, also referred to the SOX family, comprises 20 highly conserved transcription factors that play important roles in the development of prostate cancer [13]. These transcription factors are defined by a conserved signature sequence in the high-mobility group (HMG) DNA-binding domain (DBD) [14], [15]. SOX4 is a 47-kDa protein is highly conserved in vertebrates and its clinical importance has gained increasing attention in recent years, with numerous reports suggesting that SOX4 may contribute to tumor progression [16], [17]. Increased SOX4 expression is found in tumors of the bladder, prostate, and colon, and with non-small-cell lung tumors [18]–[21]. Deregulated expression of SOX4 has been correlated with increased cancer cell proliferation, cell survival, inhibition of apoptosis and tumor progression in gastric cancer [22]. Its over-expression has also been related to poor prognosis in the clinics and it is a marker to predict the outcome of patients with gastric cancer [23].

RETRACTED

However, until recently, it is unclear that whether H. pylori infection can induce SOX4 expression through down regulating miR-204. Thus, we performed our study to further investigate the role of miR-204 and SOX4 in H. pylori induced carcinogenesis.

## Materials and Methods

### Clinical Samples

Patients with or without H. *pylori* infection had undergone gastroscope at The First Affiliated Hospital of Nanjing Medical University, Jiangsu Province, China from March 2012 and December 2013. Samples taken from the 250 patients (150 noncancerous patients and 100 tumor patients) were collected, and were identified positive when rapid urease test was positive. These selected patients were also confirmed by ^13^C breath test. Noncancerous patients were classified into superficial gastritis, atrophic gastritis and dysplasia according to the pathologic classification. This protocol was approved by the Ethical Committee of the first affiliated hospital of Nanjing Medical University, and every patient had written informed consent.

### Cell culture

SGC-7901/MKN45 gastric cancer cell lines (purchased from ATCC) were cultured in RPMI-1640 medium supplemented with 10% fetal bovine serum (FBS) (Gibico) and penicillin (100 U/ml). Cells were cultured at 37°C in a humidified atmosphere with 5% CO_2_.

### Bacterial culture and infection model

H. pylori was inoculated into the plate and cultured at 37°C in a microaerophilic atmosphere with 5%O_2_, 10%CO_2_ and 85%N_2_. After 3 days, the bacterial was resuspended in RPMI-1640 medium without FBS and infected cells in a MOI of 100. Cells were then harvested after 48 h of infection.

### Isolation of total RNA and Quantitative RT-PCR

Total RNAs were extracted from collected tissues and cell lines using Trizol (Tarkara, Japan) and then both miRNA and mRNA were reverse transcribed to cDNA. The reverse transcription was performed by using reverse transcription kit (Takara, Japan). The expression of mature miRNAs and potential target genes were measured by qRT-PCR with SYBR Green PCR Kit (Takara) on Applied Biosystems StepOne-Plus Real-Time PCR System and human U6 RNA was amplified as an internal control. The relative expression ratio of miR-204 was calculated by the 2^−ΔΔCT^ method. PCR reactions were performed with the following primers: for hsa-miR-204, forward, 5′-CAUCUUCCAGUACAGUGUUGGA-3′ and for U6, forward, 5′-CTCGCTTCGGCAGCACA-3′. Relative expression levels of SOX4 mRNA were examined by SYBR Green real-time PCR (RT-PCR) and normalized to GAPDH. The primers for SOX4 were forward, 5′ AGCCATCTCGGAGGAATA 3′ and reverse, 5′ CAGACAACCGGCCTTTAT 3′; and for GAPDH, forward, 5′-CGTGGGCCGCCCTAGGCACCA-3′ and reverse, 5′-TTGGCTTAGGGTTCAGGGGGG-3′. RT-PCR was performed by using the ABI 7500 Fast Real-Time PCR system (ABI, CA, USA).

RETRACTED

### Immunohistochemistry

Tissues were fixed in 4% paraformaldehyde and cut from paraffin block to 5 µm thickness. After dewaxing with xylene and rehydration with a graded series of ethanol, slides were heated in the autoclave for three minutes using citrate sodium buffer (PH 6.0) and incubated with the antibody SOX4 (Cell signaling Technology) at 4°C overnight. Blocking serum or antibody dilution buffer was used as negative controls. The antibodies utilized before were the same as for Western blot analysis. Photographs were taken by microsope (Nikon, ECLIPSE 50i). The number of positive staining cells showing immunoreactivity of SOX4 in ten representative microscopic fields was counted, and the percentage of positive cells was also calculated. The percentage scoring of immunoreactive tumor cells was described as follows: 0 (0%), 1 (1–10%), 2 (11–50%), and 3 (>50%). The intensity was scored as follows: 0 (negative), 1 (weak), 2 (moderate), and 3 (strong). The expression level of SOX4 was measured by multiplying the percentage and the intensity score. High expression samples means tumors with a multiplied score exceeding 4 while the others were considered to be low expression.

### Cell proliferation assasy

Cell proliferation was examined using water-soluble tetrazolium salt assay using the Cell Counting Kit-8 (Dojindo, Kumamoto, Japan). In short, cells (1.5×10^3^/well) were seeded in 96-well culture plates in triplicate and incubated for 4 days at 37°C/5% CO2 in a humidified incubator. Viable cells were quantified at each 24 h interval by measuring OD450 using microplate reader (Epoch; BioTek, Winooski, VT).

RETRACTED

Cells (2×10^6^) were fixed with 75% ethanol at 4°C overnight and then washed with cold PBS and treated with RNaseI, followed by staining with propidium iodide for 30 min in dark. Cell cycle analysis was then performed by flow cytometry (FACSCalibur; Becton Dickinson, Sparks, MD).

Cells were trypsinized and plated on 6-well plates (500 cells/well) and cultured for 2 weeks. The colonies were stained with 1% crystal violet for 30 min after fixation with 4% paraformaldehyde for 30 minutes. The number of colonies, defined as >50 cells/colony were counted. Three independent experiments were performed. The data was calculated using paired t test.

### Cell migration assay (wound-healing)

A wound-healing assay was used to assess the ability of tumor cell motility. Briefly, cells (1*10^6^/well) were seeded in six-well plates, cultured overnight, and transfected with miR-204 mimics or inhibitor, pcDNA-SOX4 or pcDNA-NC. On reaching confluence, the cell layer was scratched with a sterile plastic tip and then washed with culture medium twice and cultured again for up to 48 with serum-reduced medium containing 1% FBS. The gap closure was measured and the data were summarized based on sextuple assays for each experiment.

### Cell invasion assay

Cell invasion activity was assessed using cell culture inserts coated with basement membrane matrix (BD Biosciences, Bedford, MA) according to the manufacturer's instruction. Briefly, a total of 1×105 cells in 0.2 ml serum-free RPMI-1640 medium were seeded on a Transwell apparatus. RPMI-1640 containing 10% FBS (600 µl) was added to the lower chamber. Following incubation of the cells for 24 h at 37°C in a 5% CO2 incubator, cells on the top surface of the insert were removed by wiping with a cotton swab. The cells that invaded to the bottom surface of the insert were fixed in the 100% pre-cooling methanol for 30 min, stained in 0.5% crystal violet for 30 min, then rinsed in PBS and subjected to microscopic inspection. Cells were counted under microscope in five random fields and the relative invasion and migration were interpreted as the average number of cells ± standard deviation per field.

### Western blotting

Total proteins were prepared and quantified using a protein assay (BCA method, Thermo, USA). Proteins were fractionated by sodium dodecyl sulfate polyacrylamide gel electrophoresis (SDS-PAGE) transferred to polyvinylidene fluoride (PVDF) membrane, blocked in 5% dry milk at room temperature for 1 hour and immunostained with antibodies at 4°C overnight using anti-SOX4 (1∶1000, CST, USA), anti-N-cadherin (1∶1000, CST, USA) and anti-E-cadherin (1∶1000, CST, USA). Anti-GAPDH (1∶5000, sigma,USA) was used as a loading control. Results were visualized through a chemiluminescent detection system (Pierce ECL Substrate Western blot detection system, Thermo, Pittsburgh, PA) and then exposed in Molecular Imager ChemiDoc XRS System (Bio-Rad, Hercules, CA).

RETRACTED

### Plasmid construction

Prediction of miR-204 binding sites was performed using TargetScan software (http://www.targetscan.org). 3′-UTR sequence of SOX4 which was predicted to interact with miR-204 or a mutant sequence with the predicted target sites were inserted into the KpnI and SacI sites of pGL3 promoter vector (Invitrogen). They were named pGL3-SOX4 and pGL3-SOX4-mut. The cells were plated onto 6-well plates and were transfected with 100 ng of pGL3-SOX4 or pGL3-SOX4-mut, and miR-204 mimics (50 nM) by using Lipofectamine 2000 (Invitrogen Corp, CA, USA). We normalized the differences in transfection efficiency by co-transfecting a Renilla luciferase vector pRL-SV40 (5 ng).

SOX4 gene was synthesized (purchased from Genscript, Piscataway, NJ) with restrictive digestion using Mlu I and subcloned pLV-GFP plasmid, and named pLV-GFP-SOX4. Recombinant lentivirus was generated from 293T cells using calcium phosphate precipitation. SGC-7901 cell lines were transfected with lentivirus using polybrene (8 ug/ml).

### Luciferase activities analysis

Cells were cultured in 24-well plates and transfected with 0.2 µg of either wide-type or mutant pGL-SOX4 plasmid containing firefly luciferase, together with 0.01 µg of the pGL-SOX4 vector (Invitrogen) containing renilla luciferase and 1 µg oligonucleotides. Transfection was performed using Lipofectamine 2000 reagent (Invitrogen). Relative luciferase activity was calculated 48 h post-transfection by the Dual Luciferase Reporter Assay (Promega). All transfection experiments were conducted in triplicate and repeated three times independently. Data are expressed as the mean ±SD.

### Statistical analysis

Student's t-test or one-way analysis of variance was used for statistical analysis when appropriate. All statistical analyses were performed using the SPSS 17.0 (SPSS, Chicago, IL). A two-tailed value of P<0.05 was considered statistically significant.

## Results

### MiR-204 is aberrantly down-regulated in *H. pylori* positive tissues and cells

The expression of selected miRNAs according to previous microarray data [10] were detected in 75 pairs of H. pylori positive and negative normal tissues, and 50 pairs of H. pylori positive and negative tumor tissues by real-time PCR. We found that miR-204 was one of the most significant miRNAs down-regulated upon H. pylori infection (Figure S1A, Figure 1A, B). In addition, miR-204 was expressed at lower levels in more severe gastritis (Figure 1C). We further compared its expression in tumor tissues with normal tissues, regardless of H. pylori status and found that miR-204 was expressed significantly lower in tumors (Figure S1B). We divided the patients with tumor according to different TNM stages and T2-T4 and M1 patients expressed significantly lower miR-204 than T1 and M0 patients (Figure S1C, S1D). We also examined miR-204 expression in cells infected with H. pylori and we found that the expression of miR-204 was significantly lower in multiple H. pylori infected cells than control (Figure 1D, Figure S1E).

RETRACTED

**Figure 1:** MiR-204 is down-regulated in H. Pylori positive patients. (A) The expression levels of miR-204 in human H. Pylori positive tissues and normal tissues relative to U6 were determined by qRT-PCR. (B) The expression levels of miR-204 in H. pylori positive and negative tumor tissues. (C) The expression levels of miR-204 in CG,CAG and dysplasia in H. pylori positive tissues and H. pylori negative tissue. (D) The expression levels of miR-204 in H. pylori infected cells. (*p<0.05).

### MiR-204 suppresses the migration/invasion and proliferation of gastric cancer cells in SGC-7901 and MKN-45 cells

We transfected SGC7901 and MKN45 cells with hsa-miR-204 mimic/inhibitor oligonucleotides and examined the effects on cellular proliferation and migration/invasion. Firstly, we performed qRT-PCR to verify the efficacy of transfection, as indicated in Fig. 2A, transfection of cells with miR-204 mimics/inhibitor showed significantly increase/decrease of miR-204 expression compared with their negative control (NC/iNC). Wound healing assay showed that over-expression of miR-204 could suppress cell migration, while its knockdown induced cell migration, with significant closer gap than control (Figure 2B). Consistently, Matrigel invasion assay also showed that over-expression of miR-204 attenuated cell invasion, whereas knockdown of it could reverse the affection (Figure 2C). We also performed MTT assay and found that the growth rate of cells transfected with miR-204 inhibitor was significantly increased compared with controls while cells with miR-204 mimics was showed the different (Figure 3A, B). We also examined whether the cell cycle would be affected by the knockdown/over-expression of miR-204 using fluorescence-activated cell sorting (FACS) analysis of propidium-iodide–stained cells. Knockdown of miR-204 resulted in a significant increase in the percentages of cells in the G2 phases while over-expression showed the opposite effect (Figure 3C). Colony formation assays revealed that inhibition of miR-204 significantly increased the growth rate of cell lines (Figure 3D). We also compared cell functions of transfecting with miR-204 mimics with mimics and H. pylori infection. We found that miR-204 mimics could suppress cell migration, invasion and proliferation upon H. pylori infection (Figure S2). These results together showed that down-regulation of miR-204 induced by H. pylori infection promote migration/invasion and proliferation of the gastric cancer cell line in vitro.

RETRACTED

**Figure 2:** Effects of miR-204 expression on cell invasion. (A) MiR-204 level in cells transfected with miR-204 mimics, miR-204 inhibitor, negative control (NC) and inhibitor negative control (iNC). The result was validated by real-time PCR. (B) The images photographed at 0 h (upper) and 24 h (lower) post-wounding were shown at magnification of x200. C. Cells were treated with miR-204 mimics, miR-204 inhibitor, NC and iNC for 24 h. The representative images of invasive cells at the bottom of the membrane stained with crystal violet were visualized as shown. The quantifications of cell migration were presented as percentage migrated cell numbers. All experiments were performed in triplicate and presented as mean ±SD. * indicates significant difference compared with control group (P<0.05). Every independent experiment was performed 3 times.

**Figure 3:** Effects of miR-204 expression on cell proliferation. (A) Cells transfected with miR-204 inhibitor and viabilities were determined with CCK-8 assay. (B) Cells transfected with miR-204 mimics and viabilities were determined with CCK-8 assay. (C) Effects of miR-204 mimics or inhibitor on cell cycle of gastric cancer cells by flow cytometry. (D) Colony assay after cells transfected with miR-204 mimics and inhibitor. (*p<0.05).

### MiR-204 up-regulated SOX4 expression in gastric cancer

We identified the downstream targets of miR-204 by computational prediction to elucidate the mechanisms by which miR-204 suppressed gastric cancer cell invasion. Among hundreds of genes predicted by online miRNA target prediction website (starBase, http://starbase.sysu.edu.cn/), we forcused our attention on SOX4. SOX4 had been reported to regulate gastric cancer progression and EMT or act as an underlying functional target of miR-204. To identify the prediction, through qRT-PCR and immunohistochemistry, we found that SOX4 was up-regulated in H. pylori positive tissues. Its expression was also higher in CAG than CG in H. pylori positive tissues. (n = 75, p<0.05; Figure 4A–C), which was inversely correlated with miR-204. Using Pearson's correlation analysis of SOX4-miR-204 mRNA expression, we obtained a statistically significant inverse correlation (Figure S3A, R = −0.849, P = 0.002). Using immunohistochemistry, we also discovered that SOX4 expression was significantly associated with gastric histology (p<0.05; Table 1). In vitro, we also found that SOX4 mRNA and protein level were up-regulated in gastric cancer cells infected by H. pylori (Figure S3B, S3C). We then determined the expression of SOX4 in response to the changes in miR-204 expression. Western blot and qRT-PCR assays showed that over-expression of miR-204 could significantly down-regulate the mRNA and protein expression of SOX4, while the effect of knockdown of miR-204 was the opposite (Figure 3D). We also found that the expression of EMT markers, N-cadherin and E-cadherin, was also changed related to miR-204 expression (Figure 4E), which suggested that miR-204 could affect the EMT process.

RETRACTED

**Figure 4:** Up-regulation of SOX4 in H. pylori positive tissues. The mRNA levels of SOX4 relative to GAPDH in human H. pylori positive tissues (A) including CG and CAG and normal tissues (B) were evaluated by qRT-PCR. Data were presented as scattergram of the median. * Significantly different compared with that of control (P<0.05). (C) SOX4 protein expression in H. Pylori positive and negative tissues was detected by Immunohistochemical staining. (D) SOX4 protein and mRNA levels in cells transfected with negative control (NC), miR-204 mimics; miR-204 inhibitor and iNC were analyzed through Western-blotting and qRT-PCR. GAPDH was used as a loading control. Average values of integrated optical density (IOD) were assessed by analyzing five fields per slide and recorded in the histogram. (E) E-cadherin and N-cadherin protein levels in cells transfected with negative control (NC), miR-204 mimics; miR-204 inhibitor and iNC were analyzed through Western-blotting. GAPDH was used as a loading control. Data are represented as mean±SD. * indicates P<0.05.

**Table 1:** Expression level of SOX4 in Helicobacter pylori positive tissues.

Factor	Sample N = 75	SOX4 expression (immnohistochemistry)		P value
		Low	High	
**Gender**				0.773
**Male**	42	15	27	
**Female**	33	11	22	
**Age(years)**				0.521
** <40**	34	14	20	
** ≥40**	41	12	29	
**Histology**				<0.05*
**CG**	34	15	19	
**CAG**	36	12	24	
**Dysplasia**	5	1	4	

CG: chronic gastritis; CAG: chronic atrophic gastritis;

*indicates P<0.05;

### SOX4 is a direct target gene of miR-204 in gastric cancer cells

Though SOX4 has been regarded as a direct target of miR-204, it is unclear whether miR-204 can directly recognize the 3′-UTR of SOX4 mRNA. According to the predicted target site from Targetscan, we cloned the 3′-UTR fragment containing the predicted site into the pGL3 luciferase reporter vector (pGL3-SOX4). The 3′-UTR fragment with mutated sequence within the predicted target site was also cloned as a control (pGL3-SOX4-mut). The results showed that co-transfection with miR-204 mimics and the pGL3-SOX4 vector decreased luciferase activity in SGC-7901 cells. However, miR-204 mimics did not have the effect on luciferase activity when the cells were transfected with pGL3-SOX4-mut vector (Figure 5). These data suggested that SOX4 gene was one of the direct targets of miR-204.

RETRACTED

**Figure 5:** Effects of miR-204 on SOX4 expression by luciferase reporter assay. The potential miR-204 binding site at the 3′-UTR of SOX4 mRNA was computationally predicted by Targetscan. Cells were co-transfected with miR-204 mimics (or negative control) with pGL3-SOX4 (or pGL3-SOX4-mut) vector. Luciferase activity was normalized by the ratio of firefly and Renilla luciferase signals. * indicates P<0.05.

### Over-expression of SOX4 has the effect of miR-204 on gastric cancer cells invasion

To determine SOX4 as the functional effector of miR-204 in gastric cancer invasion, we over-expressed SOX4 by transfecting with lentivirus and examined its effects in gastric cancer cells. Over-expression of SOX4 in the cell line was confirmed by western blotting (Figure 6A). We also found that E-cadherin was down-regulated while N-cadherin was up-regulated after pLV-SOX4 transfection. Through wound healing and the Matrigel invasion assay, we then discovered that the over-expression of SOX4 significantly promoted cells migration and invasion (Figure 6B and 6C). In order to further demonstrate that miR-204 induced the loss of SOX4 suppressed proliferation and invasion of gastric cancer cells, cells were transfected with miR-204 mimics and SOX4 over-expression vector together and the results showed that the suppression of migration, invasion and proliferation by miR-204 was attenuated (Figure S4).

**Figure 6:** Effects of over-expression of SOX4 by transfecting with lentivirus on cell invasion. (A) SOX4, N-cadherin and E-cadherin protein expression were analyzed by Western blotting in cells by transfecting with lentivirus, control plasmid, and Mock. GADPH was shown as internal control. (B) Wound healing assay of these images at 0 h (upper) and 24 h (lower) post-wounding were shown at magnification of x200. (C) SOX4 over-expressed and NC groups were respectively stained. The representative images of invasive cells at the bottom of the membrane stained with crystal violet were visualized as shown. The quantifications of cell migration were presented as percentage migrated cell numbers. All experiments were performed in triplicate and presented as mean ±SD. * indicates significant difference compared with control group (P<0.05). Every independent experiment was performed 3 times.

RETRACTED

## Discussion

Gastric cancer is a worldwide disease with a high incidence, especially in Southeast Asia [21]. The 5-year survival rate for gastric cancer is quite low. Some of the gastric cancer patients were H. pylori related. Therefore, it is necessary to thoroughly investigate the pathogenesis and develop new targeted treatments for H. pylori related gastric cancer.

MiRNAs are a large family of gene regulators that negatively regulate their target mRNAs in a sequence-specific manner. miRNAs may also function as tumour suppressors or oncogenes [22]. Recent evidence suggested that miRNAs play essential roles in multiple biological processes related to cancer, including cell differentiation, proliferation, tumorignesis, angiogenesis, invasion and metastasis [23]. MiR-204 has been reported to function as a tumor suppressor and low-level expression of miR-204 is associated with a poor prognostic phenotype in patients with cancer [24], [25]. However, there were few studies investigating miR-204 function in H. pylori related gastric cancer. Here, we were the first to present evidence that miR-204 was significantly down-regulated in H. pylori positive tissues (normal and tumor tissues) and that over-expression of miR-204 suppressed SOX4 protein expression and the growth of cells derived from gastric tumor.

We first quantified the expression of miR-204 in H. Pylori infection tissues and controls and we found that the miR-204 expression is significantly lower in H. Pylori infected patients. We also found that the expression is related to the histology of the patients, that is, the expression of miR-204 is significantly lower in H. Pylori positive patients with chronic atrophic gastritis than chronic non-atrophic gastritis. This expression pattern showed that possibility that miR-204 is related to different kinds of gastritis and the more severe the patients were, the lower the expression of miR-204 was. Based on the miR-204 expression level, we chose SGC-7901 and MKN45 cells for the subsequent gain-of-function and loss-of-function studies, respectively. The results suggest that down-regulation of miR-204 in gastric cancer cell is related to its progression. Although a large number of human miRNAs have been reported, many of their mRNA targets remain unidentified [9]. In this study, we used a combined bioinformatics and experimental approach to identify that SOX4 are the functional downstream target of miR-204.

SOX4 is over-expressed in various cancers and was closely correlated with tumor invasion and metastasis [16]–[19]. It is also one of members of EMT-transcriptional inducers [26]. EMT is a key developmental program that is often activated during cancer progression and may promote resistance to therapy [27]. Zhang et al [20] showed that overexpression of SOX4 in human mammary epithelial cells led to the acquisition of mesenchymal traits, and enhanced cell migration and invasion. Furthermore, SOX4 positively regulated the expression of known EMT inducers and activated the TGF-β pathway to contribute to EMT [28]. To date, EMT is an attractive target for therapeutic interventions, provides a new basis of the progression of carcinoma towards dedifferentiated and more malignant states [29]. Our study firstly showed that H. pylori infection induced miR-204 down regulation could lead to gastric cancer by EMT process.

RETRACTED

To conclude, our evidence indicated that miR-204 was down-regulated, while SOX4 was up-regulated in H. Pylori infection and gastric cancer. Ectopic miR-204 expression decreased SOX4 expression at the mRNA and protein levels in the gastric cancer cell line. We also demonstrated that miR-204 was directly bound to the 3′-UTR of SOX4. MiR-204 expression inhibited EMT via repression of SOX4. Furthermore, the miR-204-EMT pathway that we identified may be exploited in a therapeutic approach for the treatment of H. Pylori related cancers.

## Supporting Information

Figure S1 (A) The expression of 5 miRNAs in H pylori positive and negative tissues was detected by qRT-PCR. (B) The expression levels of miR-204 in tumor and control tissues. (C) The expression levels of miR-204 according to TNM stages. (D) The expression level of miR-204 in three kind of H. pylori infected cells. (*p<0.05).
(TIF)

Figure S2 **Cells transfected with miR-204 mimics and mimics with H. pylori infection and (A) viabilities were determined with CCK-8 assay (B) The images photographed at 0 h (upper) and 24 h (lower) post-wounding were shown at magnification of x200 (C) The representative images of invasive cells at the bottom of the membrane stained with crystal violet were visualized as shown.** (*p<0.05).
(TIF)

Figure S3 (A) The relative mRNA expression of miR-204 and SOX4, normalized with U6 and GAPDH, was assessed in 15 specimens of H. pylori positive and negative tissues by qRT-PCR. (B) An inverse correlation of SOX4 and miR-204 expression levels was examined (R = -0.920, P = 0.001). (C) The expression of SOX4 mRNA was determined by qRT-PCR in H. pylori infected cells. (D) The expression of SOX4 protein level was determined by western blot in H. pylori infected cells. (*p<0.05).
(TIF)

Figure S4 **Cells transfected with miR-204 mimics and mimics with pLV-SOX4 and (A) viabilities were determined with CCK-8 assay (B) The representative images of invasive cells at the bottom of the membrane stained with crystal violet were visualized as shown.** (C) The images photographed at 0 h (upper) and 24 h (lower) post-wounding were shown at magnification of x200 (*p<0.05).
(TIF)
